This article has been retracted.

# The Effects of Elgucare on Degenerated Intervertebral Disc-Induced Low Back Pain and Disc Regeneration: A Clinical Trial

**DOI:** 10.1155/2021/5824956

**Published:** 2021-11-08

**Authors:** Wen-Cheng Lo, Yu Ting Chen, Chen Ching Chen

**Affiliations:** ^1^School of Medicine, College of Medicine, Taipei Medical University, Taipei, Taiwan; ^2^Department of Neurosurgery, Taipei Medical University Hospital, Taipei, Taiwan; ^3^Department of Surgery, School of Medicine, College of Medicine, Taipei Medical University, Taipei, Taiwan; ^4^Research and Development of DC Botanical Biotechnology CO., LTD, LDY Chinese Medicine Hospital, New Taipei City, Taiwan; ^5^DC Botanical Biotechnology CO., LTD, LDY Chinese Medicine Hospital, New Taipei City, Taiwan

## Abstract

**Introduction:**

Chronic low back pain (LBP) has a wide range of causes. However, most cases are induced by degeneration of the lumbar intervertebral discs (IVDs), and the aching caused by local compression of the affected region has considerable impacts on quality of life. This clinical trial investigated the use of Elgucare, a Chinese herbal formula, as a food supplement to reduce the pain of patients with LBP induced by degeneration of the lumbar IVDs.

**Methods:**

The study assessed patient subjective quality of life, functional limitations caused by LBP, and variations in pain. The assessment was done through the visual analogue scale (VAS) and effects on lumbar IVD thickness, water content, and bone mineral density (BMD). These parameters were evaluated before and after the administration of Elgucare or a placebo, one of which was taken by each participant for a 12-month period.

**Results:**

Elgucare reduced the patients' mean VAS pain score by 2.25 points and improved their mean LBP-hampered mobility as assessed by the Roland-Morris Questionnaire by 5.17 points. The results of another questionnaire indicated that Elgucare slowed the LBP-induced deterioration of patients' quality of life, while objective assessment indices obtained through X-ray and magnetic resonance imaging showed that the height and water retention of their IVDs were increased. However, the BMD results showed no improvements.

**Conclusions:**

Elgucare can increase the water retention and height of IVDs and reduce LBP, thereby enhancing quality of life. Therefore, Elgucare can potentially be used as a clinical supplement.

## 1. Introduction

Low back pain (LBP) is often induced by intervertebral disc degeneration (IDD), which is a major disease of aging [1, 2]. Intervertebral disc (IVD) tissues are located between IVD bodies and are composed of annulus fibrosus (AF) and nucleus pulposus (NP) tissues. NP tissues retain high water content and provide a crucial buffer function of maintaining IVD height and spinal joint mobility [3]. Although the water content of NP tissues in children is typically greater than 80%, it decreases with age, dropping as low as 70% in older individuals, and this loss of water content is a major cause of IDD [4].

Relatedly, IDD usually occurs in adult individuals, and as IDD progresses, the load surrounding AF tissues increases, causing the IVDs to collapse, which in turn generates direct friction in the vertebral body and induces the growth of bone spurs and/or LBP [5–7]. Once IDD occurs, irreversible deterioration continues. The causes of chronic LBP can be extremely diverse, but lumbar IDD is one major cause of chronic LBP. This is because of the resulting impaired ability of the spine to distribute pressure, which again is caused by dehydration and deterioration of the IVDs [7]. This is also called discogenic LBP. Its diagnosis is based on the presence of chronic LBP (sometimes accompanied by radicular pain) and positive provocative discography [8]. Studies have indicated that evidence of IDD can be identified by magnetic resonance imaging (MRI) in approximately 30% of asymptomatic adult test subjects over 30 years old, while similar changes can be identified in almost all individuals over 60 years old [9–11].

The major cause of long-term chronic LBP is degeneration of the IVDs, which, as indicated above, typically worsens with age [10, 11]. As the patient ages, the number of cells in the NP and AF decreases, the ability of the NP to retain water is reduced, and the AF gradually loses moisture and displays fibrosis. This decreases the IVD height under loading and affects the uniform distribution of pressure, often resulting in localized stresses [5, 6, 12].

From the perspective of the tissue structure, the posterior edge of the AF is a region of loose fiber and poor stability. It is located next to the posterior longitudinal ligament (PLL), which is the lumbar tissue with the most dense distribution of pain nerves [3]. Nociceptors are mainly distributed in the peripheral area of the posterior side of the lumbar IVDs [13]. The sensation of pain is transmitted through the dorsal root ganglia (DRG) [14]. Pain in LBP patients may be caused by the inability of the degenerated IVDs to withstand unstable spine movements, which thus cause pain through the release of various inflammatory proteins [13, 15]. As deterioration progresses, the symptoms worsen until the IVDs become completely dehydrated. At this stage, the pain begins to be reduced, but symptoms of nerve compression remain there [16, 17].

Currently, there are various conventional treatments for LBP. For example, drug therapies such as aspirin, nonsteroidal anti-inflammatory drugs (NSAIDs), oral steroids, and narcotic analgesics can be used for pain relief, although such therapies often come with various side effects [18]. Meanwhile, physical therapies such as hot packs, electrical stimulation, and exercise may also be employed [18–20].

Chemonucleolysis, which consists of the percutaneous injection of chymopapain or collagenase into the NP to dissolve partial IVDs, thereby reducing the pressure exerted on the nerve root and relieving pain and numbness, has also been used [21]. However, it is not applicable for cases of chronic or lumbar spine disorders or ruptured discs, and it can trigger severe allergic reactions [22, 23]. Therefore, it is only rarely performed at present. In terms of surgical treatments, disc removal is commonly performed, while cage interbody fusion or artificial disc replacement surgeries may be required in severe cases. However, artificial disc implants consist of polymer-metal composites and are very costly, and such implants can also cause pain, discomfort, and other side effects due to poor biological compatibility [24]. With regard to fusion surgeries, meanwhile, the surgical process can cause excess bleeding and damage normal spinal structures, extending the postoperative healing period to half a year or more [25].

Improvement is usually limited when patients with compressed nerves or tissues, due to severe spinal cartilage degradation, are treated using the aforementioned methods. Current studies on clinical treatments have shown that younger patients with symptoms for less than six months have exhibited improved outcomes [26]. However, 80% of patients recovered on their own because the herniated cartilage will eventually dehydrate and shrink, no longer compressing the nerves and thus enabling the condition to heal naturally [27]. The primary conventional surgery, again, is IVD removal, while fusion and screw fixation are performed, when needed, to fuse and fix the vertebrae. This provides adequate short-term effects but hampers the mobility of the fixed segments, resulting in stiff lumbar movements and restrained twisting, bending, and stretching movements. The restrictions also increase the stresses on adjacent IVDs, predisposing patients to herniation of the adjacent segments and hence leading to adjacent segment disease (ASD) [28]. Therefore, postfusion patients are extremely likely to undergo surgery again within a few years. Alternatively, a newer method of neurological decompression coupled with nonfusion spinal surgery has been developed and has demonstrated promising results in recent years, but its long-term effects have yet to be observed [29].

The compatibility theory of traditional Chinese medicine emphasizes the tendency of natural herbs to promote self-healing. The same theory was adopted in the development of Elgucare, the Chinese herbal formula investigated in this study. Various medicinal herbs were included in the formula based on their ability to regulate physiological functions, enhance physical strength, promote metabolism, maintain health, and supply nutrients [30]. In addition to those effects, the formula was expected to eliminate obstructions in microcirculation and thereby improve spinal pain resulting from local hypoxia, thus alleviating soreness and numbness caused by vertebral deterioration [31].

Therefore, the current study was conducted in order to determine the effects of Elgucare in LBP patients, particularly in terms of pain relief.

## 2. Materials and Methods

### 2.1. Study Protocol

The objective of this clinical trial was to assess the effects of Elgucare on the subjective quality of life, functional limitations caused by LBP, pain as assessed through the visual analogue scale (VAS), and lumbar IVD thickness, water content, and BMD of patients with chronic LBP induced by lumbar IVD degeneration. To assess the effects of Elgucare on these parameters, the study participants were randomly assigned into two groups: an Elgucare group that was treated with Elgucare and a control group that received a placebo. The Elgucare group ingested three 500 mg capsules of Elgucare twice per day for 12 months, while the control group ingested three 500 mg placebo capsules twice per day for 12 months. The study parameters were evaluated before, during, and after the 12-month treatment period.

### 2.2. Evaluation Indices

The primary evaluation indices were the VAS, the Roland-Morris Questionnaire (RMQ), and the Short Form 36 Health Survey Questionnaire (SF-36), which were used to evaluate and compare the patients' pain levels, improvements in LBP, and improvements in quality of life, respectively. These questionnaires were administered once before the 12-month treatment period and then at subsequent visits made every month for the following 12 months. The secondary evaluation indices included MRI scans, X-rays, and BMD data. The BMD data were used to assess and compare the BMD levels of the Elgucare and control groups, while the X-rays were used to examine and compare the subjects' L-spine anteroposterior (AP) values, and the MRI images and the T2-weighted signals of the MRI images were used to evaluate and compare the disc height and water content, respectively, at the core of the participants' IVDs. Furthermore, blood chemistry tests were conducted to evaluate the patients' levels of calcium (Ca), sodium (Na), potassium (K), chloride (Cl), blood glucose (GLU), uric acid (UA), blood urea nitrogen (BUN), creatinine, SGOT/AST, and SGPT/ALT. The MRI and X-ray exams were conducted shortly before the start of the 12-month treatment period and then at 6, 9, and 12 months within the treatment period, while the BMD exams were conducted before the treatment period and at 6 and 12 months during the treatment period. The blood chemistry tests were conducted before the treatment period and then every two months during the treatment period.

### 2.3. Inclusion and Exclusion Criteria

The criteria for inclusion in the study were as follows:

1. Age ≥ 20 and ≤50 years
2. A diagnosis of long-term LBP caused by lumbar IVD degeneration and occasional sciatica confirmed by a professional orthopedist

The exclusion criteria were

1. a diagnosis of rheumatoid arthritis, ankylosing spondylitis, gouty arthritis, osteoarthritis of the knee, scoliosis, spondylolisthesis, myeloma, or neurofibroma
2. a diagnosis of osteoporosis with vertebral fracture that was treated with surgical artificial bone cement reinforcement
3. a spinal injury caused by accident, external force, or degeneration that was treated with spinal surgery
4. a diagnosis of chronic disease, autoimmune disease, thrombasthenia, severe hypertension, diabetes, or cancer
5. an allergy to traditional Chinese medicine
6. pregnancy or lactation
7. gastrointestinal bleeding within the past four weeks, or
8. taking medications other than acetaminophen

In addition, the eligible patients were required to not be diagnosed as having muscle atrophy or other neurological symptoms and had to require no immediate aggressive surgical treatment (i.e., due to severe radiculopathy or cauda equina syndrome).

Each patient considered for inclusion in the study was fully informed of his or her rights before his/her informed consent was obtained. Approval for the study was sought and received from the independent review board of a university hospital in Taiwan that served as the setting for the research.

### 2.4. Statistical Analysis

The effects of the intervention on all of the dependent variables (i.e., the VAS score, RMQ total score, eight domains of the SF-36, X-ray- and MRI-related parameters, and *t*-score of BMD) were assessed using a generalized estimating equation (GEE). Each GEE model included the main effects of intercept, group (1 = Elgucare; 0 = control), and measurement (time points as a categorical variable), as well as two-way interactions of “group × measurement.” A significant two-way interaction indicated a significant difference in the change from the baseline to a later period of time between the two groups. In addition, the differences in each dependent variable between the Elgucare group and the control group at specific time points were also assessed using the simple main effect within the GEE model. All tests were 2-tailed, and *P* < 0.05 was considered statistically significant. No adjustment of multiple testing (multiplicity) was made in this study. Data analyses were conducted using SPSS 25 (IBM SPSS Inc., Chicago, Illinois).

## 3. Results

A total of 40 participants were enrolled, of whom 24 were enrolled in the Elgucare group and 16 were enrolled in the control group. In the Elgucare group, 10 (42%) of the participants were women, while in the control group, 5 (31%) were women. The mean ages of the experimental group and control group participants were 41.8 and 38.9 years old, respectively.

Figure 1 displays the mean VAS and RMQ total scores of each group across the different time points. These results indicate that the control group had a greater improvement in the VAS score from visit 1 to visit 2 and from visit 1 to visit 4 (both *P* < 0.05; Figure 1(a)). In addition, the VAS score of the control group at visit 4 was significantly lower than that of the Elgucare group. For the RMQ total score, no significant differences between the groups were observed at any specific period of time (Figure 1(b)).

Furthermore, no significant differences between the groups were found at any specific period of time for six domains of SF-36, namely, the physical functioning, role-physical, role-emotional, social functioning, mental health, and vitality domains (Figures 2(a)–2(d), 2(f), and 2(g)). However, the improvement in the bodily pain domain from visit 1 to visit 3 was greater in the Elgucare group than in the control group (*P* < 0.05; Figure 2(e)). Furthermore, the results indicated that the scores for the general health domain at visit 8 were greater for the Elgucare group than for the control group (Figure 2(h)).

Figure 3 shows the results for the X-ray- and MRI-related parameters. The L-spine AP values measured by X-ray at visit 1 were significantly greater for the control group than for the Elgucare group (Figure 3(a)). However, no significant difference between the two groups was observed in terms of the L-spine true lateral view values measured by X-ray, the central disc height values measured by MRI, or the T2-weighted values measured by MRI (Figures 3(b)–3(d)).

The results further indicated that the participants in the Elgucare group had significantly lower *t*-score of BMD values at the follow-up visit than did those in the control group (Figure 4).

Finally, the blood chemistry tests conducted every two months to evaluate the participants' blood levels of Ca, Na, K, Cl, GLU, UA, BUN, creatinine, SGOT/AST, and SGPT/ALT showed no noticeable changes in those levels for the Elgucare group or the control group, with the results for the Elgucare group indicating that Elgucare is a safe supplement that does not have any adverse effects on patient health.

## 4. Discussion

The VAS and the “bodily pain” domain of the SF-36 survey have long been used to measure patients' perceived levels of pain [32, 33]. In this study, both the VAS results and pain-related results of the SF-36 indicated that the participants who took Elgucare reported improved pain scores over the course of the study. Meanwhile, the RMQ, which provides self-rated health scores related to the inconveniences to daily life caused by LBP, has been extensively applied to evaluate improvements in quality of life among LBP patients [34], and the RMQ results for this study showed that Elgucare helps in improving the participants' scores regarding the direct perception of pain.

We also used objective image monitoring to evaluate the effects of Elgucare on physical parameters related to LBP. The inspection of X-ray, MRI, and other types of radiologic images is the main method used by clinical physicians to evaluate the level of degeneration in LBP patients' IVD tissues. In fact, even when a patient experiences no pain during the initial period of IDD, such images can be used to identify tissue and structural changes in the IVD [10, 11]. In IVD tissues, the production of interstitial proteoglycans can be decreased, causing dehydration within the IVD, fibrosis of the tissue, and loss of osmotic pressure within the NP tissues [35]. These are all primary contributing factors in IDD and disc height reduction and cause the NP tissue at the core of the IVDs to lose its damping ability. In the present study, therefore, we first used X-rays to examine the subjects' L-spine AP values and then used the MRI images and the T2-weighted signals of the MRI images to evaluate the disc height and water content at the core of the participants' IVDs, respectively, as these results essentially reflect the degree of IDD [9]. That said, no significant differences between the Elgucare group and the control group were observed in terms of the L-spine true lateral view values, the central disc height values, or the T2-weighted values.

Clinically, a desirable treatment for IDD must achieve at least one of the following three objectives: improvement in back pain, the reduction or reversal of IVD tissue metabolism, or the promotion of tissue growth. IVDs lack nutrient penetration, so once tissues irreversibly degenerate, external treatment is required to promote cell regeneration within the tissue and increase secretion of the tissue matrix. This is necessary to increase water retention and maintain turgor pressure within the IVDs and thereby maintain or increase IVD heights. As a result, IVD structures can be improved, inhibiting symptoms of LBP [36].

Relatedly, a clinical study by Fenty et al. indicated that MRI images can be used to examine the biochemical composition and external appearance of IVDs and thus assess the degree of degeneration [37]. The same study found that IVD heights are inversely proportional to an LBP patient's degree of pain; that is, as IVD heights decrease, the pain experienced by the patient increases. In this sense, MRI images and VAS and other pain indicator results are interrelated [37]. In the current clinical trial, the VAS and pain-related results of the SF-36 were found to be improved among the participants who took Elgucare.

Trace elements (TEs) are a crucial factor in the physiology of IVDs. Specifically, TEs can help synthesize enzymes, stimulate NP tissue matrix synthesis within IVD tissues, maintain turgor pressure within the tissue, and promote IVD health [38]. Relatedly, a number of Chinese herbal medicines and ingredients have been demonstrated to improve IDD. Liang et al. adopted an IDD rat model and found that by using the herbal medicine treatment formula, *Fufangqishe-Pill* increased type II collagen and suppressed matrix metalloproteinases (MMPs) and inflammatory factor IL-1*β*, thereby promoting tissue regeneration effects [39]. In another study, Klawitter et al. used the pure Chinese herbal medicinal extract Triptolide (TPL) in a culture model of human IVD cells and found that TPL suppressed TLR expression and MAPK activity and had anti-inflammatory effects [40]. These previous studies confirmed that effective Chinese herbal medicinal ingredients can suppress IDD and promote tissue regeneration and thus support the results for Elgucare found in the present study. That said, while the results of this study indicated that Elgucare resulted in better water retention than the placebo (which in turn may have been responsible for the better pain scores of the Elgucare treatment group), it is not clear exactly how Elgucare causes water to be retained in IVD tissues. As such, this effect of the supplement should be studied further in future research.

In summary, Elgucare can improve subjects' LBP-induced pain, thereby enhancing LBP patients' quality of life. Therefore, Elgucare can potentially be used as an effective clinical supplement.

## 5. Conclusions

The present study investigates the effects of Elugacare, a Chinese herbal medicine, on subject quality of life and its functional limitations through the clinical trial. Elgucare can increase the water retention and height of IVDs and reduce LBP, thereby enhancing quality of life. In the present trial, it was also found that Elgucare is a safe supplement that does not have any adverse effects on patient health. Therefore, Elgucare can potentially be used as a clinical supplement. Further studies are required to understand the mechanism of how Elgucare causes water to be retained in IVD tissues.

## Figures and Tables

**Figure 1:** Comparisons of VAS score (a) and RMQ total score (b) between the Elgucare group and the control group across the different time points. The red squares (for the Elgucare group) and green diamonds (for the control group) indicate the mean values, and the error bars indicate the standard errors of the means. Each ∗ indicates that the group difference in the change from baseline to the later time point was significant. † indicates that the group difference at a specific time point was significant. Abbreviations: RMQ: Roland-Morris Questionnaire; V: visit; VAS: visual analogue scale; FU: follow-up visit.

**Figure 2:** Comparisons of physical functioning (a), role-physical (b), role-emotional (c), social functioning (d), bodily pain (e), mental health (f), vitality (g), and general health scores between the Elgucare group and the control group across the different time points. The red squares (for the Elgucare group) and green diamonds (for the control group) indicate the mean values, and the error bars indicate the standard errors of the means. ∗ indicates that the group difference in the change from the baseline to the later time point was significant. † indicates that the group difference at a specific time point was significant. Abbreviations: SF: short form; V: visit; FU: follow-up visit.

**Figure 3:** Comparisons of L-spine AP (a) and L-spine true lateral view (b) values measured by X-ray and central disc height (c) and T2-weighted (d) values measured by MRI between the Elgucare group and the control group across different time points. The red squares (for the Elgucare group) and green diamonds (for the control group) indicate the mean values, and the error bars indicate the standard errors of the means. † indicates that the group difference at a specific time point was significant. Abbreviations: MRI: magnetic resonance imaging; V: visit; FU: follow-up visit.

**Figure 4:** Comparison of *t*-score of BMD values between the Elgucare and control groups across different time points. ∗ indicates that the group difference in the change from the baseline to the later time point was significant. Abbreviations: BMD: bone mineral density; V: visit; FU: follow-up visit.

## Data Availability

The data that support the findings of this study are available from the corresponding author, C.C.C., upon reasonable request.
